# An Algorithm for Time Prediction Signal Interference Detection Based on the LSTM-SVM Model

**DOI:** 10.1155/2022/1626458

**Published:** 2022-03-11

**Authors:** Ningbo Xiao, Zuxun Song

**Affiliations:** School of Electronics and Information, Northwestern Polytechnical University, Xi'an 710072, Shaanxi, China

## Abstract

Interference detection is an important part of the electronic defense system. It is difficult to detect interference with the traditional method of extracting characteristic parameters for interference generated at the same frequency as the original signal. Aiming at this special time-frequency overlapping interference signal, this paper proposes an interference detection algorithm based on the long short-term memory-support vector machines (LSTM-SVM) model. LSTM is used for the time series prediction of the received signal. The difference between the predicted signal and the received signal is used as the feature sample, and the SVM algorithm is used to classify the feature samples to obtain the recognition rate of whether the sample has interference. The LSTM-SVM model is compared with the gate recurrent unit-support vector machines (GRU-SVM) model, and the comparison results are visualized using a confusion matrix. The simulation results show that this LSTM-SVM model algorithm cannot only detect the existence of the interference signal but also can determine the specific position of the interference signal in the received waveform, and the detection performance is better than the GRU-SVM model.

## 1. Introduction

In the present study, algorithms based on deep learning are booming, and research on algorithms based on deep learning has been proposed in many fields. LSTM neural networks can better predict time series data, and various algorithms based on LSTM to predict future development are also being widely used. Natural disaster prediction is a very important application. LSTM is used to learn the spatiotemporal relationship between disasters in different locations, and this relationship is used to make predictions. Through the training of historical trajectory data, the trajectory prediction model is obtained, so that early warning can be achieved [1, 2]. In terms of health care, the use of an LSTM network to independently detect the contraction curve of an ECG or EMG signal, based on the predicted signal, provides a powerful assistant for medical staff to quickly diagnose and help patients recover [3–5]. Adopting LSTM can achieve higher accuracy than traditional mathematical models in predicting future disease trends [6]. In terms of traffic prediction, new methods for urban traffic prediction combining spectrogram analysis and LSTM have been proposed [7, 8]. Using an LSTM network, electric cars can estimate future speed in real-time to estimate the precise value of brake pressure [9]. In addition, subway passenger flow prediction using LSTM can guide passengers to effectively select departure times and transfer from station to station [10]. It is widely used in fault detection, such as image forgery detection, analyzing discriminative features between different regions by combining encoder and LSTM networks, to predict whether the image has been tampered with [11]. LSTM can provide inpainting for video frames, using convolutional LSTM-based encoders and decoders to predict missing frames [12]. LSTM can achieve a predicted quantified output of the remaining mechanical life [13].

At present, the related research involving interference detection in wireless communication is increasing day by day, and some effective algorithms have been proposed. Some of these algorithms are based on computer network protocols and detect the presence of interference signals by detecting the listening time of the carrier signal; Some algorithms analyze the signal according to the frequency domain transformation, and perform the frequency domain transformation on the signal to extract features, then analyze whether there is interference in the signal; some algorithms achieve the purpose of signal analysis by counting the mathematical characteristics of the signal and calculating the high-order statistics of the signal so as to extract the signal characteristics. Obviously, the above method belongs to the traditional interference detection method, which mainly analyzes the parameter characteristics such as the spectrum and power of the received signal, and then confirms whether there is interference. Secondly, when the signal overlaps with the interfering frequency, the eigenvalues of the interfering signal are difficult to detect [14].

Since communication signals belong to time series data, the time series prediction algorithm based on deep learning provides an idea for signal interference detection. Among them, the recurrent neural network has the characteristics of short-term memory. If the time series signal is long, it will affect the transmission of information. LSTM and gate recurrent unit (GRU) can solve short-term memory problems. Based on the existing research field, we combine LSTM and GRU with the SVM model and propose the LSTM-SVM and GRU-SVM models for signal interference detection [15].

## 2. Materials and Methods

A signal is a periodic time series data, and unknown sampling points can be predicted through the correlation between sampling points [16]. According to this feature, assuming that the training signals are all normal signals, the predicted future signals should also be normal signals. In this case, calculating the difference between the real signal and the predicted signal as the detection feature can get a good detection effect. The signal prediction problem can be solved by the LSTM network. In essence, signal prediction is a time series prediction problem with periodic characteristics. The previously received signal is used as the input, and the output is the signal at the moment you want to predict.

### 2.1. Structure of LSTM

The LSTM unit structure is shown in Figure 1. Compared with the RNN cell structure, LSTM adds a cell state to the structure. LSTM neurons consist of a forget gate, an input gate, and an output gate. The forget gate is used to determine the importance of information, the input gate is used to update the cell state, and the output gate is used to calculate the value of the hidden state.

### 2.2. Structure of GRU

The GRU unit structure is shown in Figure 2. Compared with the LSTM cell structure, the GRU reduces the cell state. The neurons of the GRU include an update gate and a reset gate [17]. The update gate is used to determine the importance of the information, while the reset gate is used to determine the proportion of retained information. Compared to LSTM, GRU has simpler neurons and therefore faster training.

### 2.3. Activation Function: Tanh, Sigmoid

The Tanh function is used to adjust the threshold of the function output. The value range is [−1, 1], as shown in Figure 3.

(1) $$\begin{array}{c} f\left(x\right)=\frac{\sinh\left(x\right)}{\cosh\left(x\right)}=\frac{1-e^{-2x}}{1+e^{-2x}} \end{array}$$

The activation function Sigmoid is similar to the tanh function, with a value range of (0, 1), as shown in Figure 4.

(2) $$\begin{array}{c} \sigma =\frac{1}{1+e^{-x}} \end{array}$$

### 2.4. Time Series Signal Forecasting

60% of the received signal is used for training datasets of LSTM and GRU. The remaining 40% of the signals, as the test dataset, are used for prediction. The eigenvalues are obtained by subtracting the test data from the predicted data. The process is shown in Figure 5 [18].

When the normal communication signal in the received signal adopts the cosine signal and the interference signal adopts the narrow-band Gaussian noise [19], the LSTM time series signal prediction is shown in Figure 6, the obtained eigenvalues are shown in Figure 7.

The first picture of Figure 6 is the original received signal. You can see that there are interference signals between 2500–3000. The second picture is the training and prediction time series of LSTM, where the first 60% is the training set, and the last 40% is the prediction value. The first picture in Figure 7 is the 40% of the received signal that needs to be predicted. The second picture is the comparison of the predicted value with the original received signal, and the third simulation plot is the eigenvalues [20].

### 2.5. Windowing of Signal Sample Values

In the detection process, when the deviation of each sampling point is used as a feature to train the SVM classifier, the difference calculated for the test dataset, especially the part containing the interference signal, contains many differences similar to the difference calculated from the normal signal points, and these points are difficult to detect. So, we add windows to the features based on the time step and detect them based on the waveforms and correlations of multiple feature points to overcome contingency. The windowing process is shown in Figure 8.

If only each sampling point were used as a feature of interference detection, the detection effect would be very poor due to the accidental error of calculating the difference. Therefore, here we select the mean value of the sampling points of each *n* continuous signal as a feature, and the method of constant translation is used to construct a complete feature of interference detection. As shown in Figure 8, the signal is windowed, the window length is “*N*,” the step length is “*S*,” and the input data is formed in time series. The value of *S* is 1, when *N* is an odd number, the *i*th eigenvalue is calculated according to formula (3), and when *N* is an even number, the *i*th eigenvalue is calculated according to formula (4).

(3) $$\begin{array}{c} V_{i\_e}=\frac{V_{i-\left(N-1\right)/2}+...+V_{i-1}+V_{i}+V_{i+1}+...+V_{i+\left(N-1\right)/2}}{N} \end{array}$$

(4) $$\begin{array}{c} V_{i\_e}=\frac{V_{i-N/2+1}+...+V_{i}+V_{i+1}+...+V_{i+N/2}}{N} \end{array}$$

### 2.6. Data Normalization Processing

The eigenvalues are normalized and preprocessed, the normalization method adopted is according to the following formula:

(5) $$\begin{array}{c} f:x⟶y=\frac{x-x_{\min}}{x_{\max}-x_{\min}} \end{array}$$

## 3. Results

In the AWGN channel environment, the sampling frequency of the received signal is 3 KHz, the center frequency of the communication signal and the interference signal is 1 KHz, and the signal power is 10 dB. The sampled signal of the received signal *r*(*t*) is *r*(*n*), as shown in formula (6).

(6) $$\begin{array}{c} r\left(n\right)=s\left(n\right)+j\left(n\right)+w\left(n\right),n=1,2,\ldots ,N \end{array}$$

In the above equation *N* is the sampling length, *s*(*n*) is the communication signal, *j*(*n*) is the interference signal, and *w*(*n*) is the Gaussian white noise.

### 3.1. Comparison of the Influence of SNR on Interference Detection

Both LSTM and GUR are set to train the first 0.6 parts of the time series of the data and test the remaining 0.4 parts at 100 training iterations. After obtaining the eigenvalues, the eigenvalues are not subjected to windowing processing, and the eigenvalues are classified in the SVM to obtain the interference detection rate. When the signal power is 10 dB, the SNR value range is 0dB–20 dB, and the step size is 2 dB, the interference detection accuracy is shown in Figure 9.

It can be seen from Figure 9 that, the difference data obtained by the LSTM and GUR time prediction models are not windowed. As the SNR increases, the detection rate of the difference signal by SVM also gradually increases.

### 3.2. Comparison of Windowing Experiments

Due to the continuity characteristics of the interference signal, taking into account the correlation between the sampling points, window processing is performed on the sampling points, which can overcome the influence of accidental errors. When the power of the signal is 10 dB and the SNR is 20 dB, the eigenvalues are processed by windowing. The window length is 1–10, the step size is 1, and the interference detection accuracy is obtained as shown in Figure 10.

It can be seen from Figure 10 that LSTM has the highest detection rate when the window length is 6, but the GRU windowing effect is not good. The detection rate is the highest when no window is added, so the window value is selected as 1.

### 3.3. Interference Detection Accuracy under the Optimal Window

The difference signal generated by the LSTM is windowed with a length of 6 and the difference signal generated by the GRU is not windowed. After normalization, it is sent to the SVM for classification. The classification result diagram is shown in Figure 11 [21].

It can be seen from Figure 11 that, when there is an interference signal, the interference detection accuracy of LSTM-SVM is 93.6%, and the interference detection accuracy of GRU-SVM is 89.6%.

### 3.4. Confusion Matrix

Since the SVM classification results cannot see the detection accuracy of each type, we use a confusion matrix to further refine the detection results. The confusion matrices for LSTM-SVM and GRU-SVM interference detection classification are shown in Figure 12 [22].

From Figure 12, it can be seen that, when there is no interference, the detection accuracy of the GRU-SVM is 100%, and that the detection accuracy of the LSTM-SVM model is 99.5%. When there is interference, the detection accuracy of GRU-SVM is 68.7%, and the detection accuracy of LSTM-SVM is 81.8%. Overall, the false detection rate of GRU-SVM is 10.4%, and the false detection rate of LSTM-SVM is 6.4%. Therefore, the eigenvalues obtained by LSTM-SVM are more conducive to detecting the presence of interference signals.

## 4. Discussion

The traditional interference detection starts from the received signal, analyzes the frequency domain characteristics of the received signal, extracts the characteristic value, and then determines whether there is an interference signal. However, when the interference signal and the communication signal have the same frequency, it is difficult to extract the eigenvalues by using the traditional method. From the perspective of the time domain, this paper adopts the LSTM model, which has good prediction ability for time series signals. The eigenvalues are obtained from the difference between the predicted signal and the received signal, which solves the problem of signal interference detection in the case of interference.

The setting of the interference signal in the experiment described in this paper is relatively ideal. The interference signal used in this paper is a partial frequency band interference signal, that is, the interference signal is generated by Gaussian noise through a narrow-band filter. You can try to use other interference signals to verify whether the experimental results in this paper are applicable.

## 5. Conclusion

Aiming at the detection of special time-frequency overlapping interference signals, an interference detection algorithm based on the LSTM-SVM model is proposed in this paper. LSTM is used for the time series prediction of received signals, and the difference between the predicted signal and the received signal is used as a feature sample. This method can still be trained using a small amount of data and can obtain better prediction performance. The eigenvalue samples are windowed, and the SVM algorithm is used to classify and detect the eigenvalue samples. The LSTM-SVM model is compared with the GRU-SVM model. The comparison results show that the interference detection accuracy of the two models increases with the improvement of the SNR. Windowing the eigenvalues can significantly improve the interference detection performance of the LSTM-SVM model, but windowing the GRU-SVM model will reduce the accuracy. Under the optimal window, the detection performance of the LSTM-SVM model algorithm is better than that of the GRU-SVM model. This algorithm, based on the LSTM-SVM model, has reference significance for the research of interference detection methods.

## Figures and Tables

**Figure 1:** Structure of LSTM.

**Figure 2:** Structure of GRU.

**Figure 3:** Activation function tanh.

**Figure 4:** Activation function sigmoid.

**Figure 5:** Block diagram of the signal prediction process.

**Figure 6:** LSTM timing signal prediction.

**Figure 7:** Eigenvalues.

**Figure 8:** Signal data windowing process.

**Figure 9:** Influence of SNR on detection accuracy.

**Figure 10:** Effect of signal windowing on detection rate.

**Figure 11:** Simulation of interference detection accuracy.

**Figure 12:** Confusion matrix of LSVM-SVM and GRU-SVM classification.

## Data Availability

The data used to support the findings of this study are available from the corresponding author upon request.
